# A Study on Exploring the Path of Psychology and Civics Teaching Reform in Universities Based on Artificial Intelligence

**DOI:** 10.1155/2022/4841387

**Published:** 2022-08-08

**Authors:** Liang Han, Jijuan Gong

**Affiliations:** ^1^School of Marxism, Chongqing College of Humanities, Science and Technology, Hechuan, Chongqing 401520, China; ^2^School of Politics and Law, Chongqing College of Humanities, Science and Technology, Hechuan, Chongqing 401520, China

## Abstract

The development of precise teaching of civics with artificial intelligence not only is the realistic need of the development of the times and technological innovation but also provides a new picture to solve the problem of the relevance of civics, so it is the inevitable requirement for the quality and efficiency of civics teaching. Curriculum Civics is an important support for the cultivation of innovation ability of college students. To effectively identify the state categories of college students' psychology and civics and to fully consider the emotional factors between teachers and college students, this paper proposes a psychological civics teaching model based on graphical convolutional neural network. First, the dialog texts of psychology and civics teaching between teachers and students are coded in sequence context using Bi-GRU to obtain discourse text representations; then, a directed graph is constructed based on the order of the dialog between teachers and students in psychology and civics teaching, and a new text representation vector for each discourse text is obtained using graph convolutional neural network; finally, the two discourse representation vectors obtained are connected, and a similarity-based attention mechanism is used. Finally, the final discourse text representation is obtained using an attention-based mechanism to perform psychological and ideological state. The proposed method is conducive to the implementation of the teaching practice exploration of organic integration of ideals and beliefs with the cultivation of innovation ability in colleges and universities.

## 1. Introduction

In the National Conference on Ideological and Political Work in Colleges and Universities, General Secretary put forward the concept of “Curriculum Civics,” emphasizing that teachers should integrate socialist core values into the whole process of teaching and educating people, so that all courses can play the role of ideological and political education, and realize the same direction of professional courses, public courses, and ideological and political theories, thus resonating and forming a synergistic effect [1–3]. To implement this teaching concept, all universities actively explore the teaching reform of curriculum thinking and politics, trying to educate people through “all courses, all aspects, all staff”; effectively respond to the development needs of “big thinking and politics” in the new era; realize the goal of curriculum thinking and politics; and achieve the goal of “establishing moral education.” During the period of accelerated social transformation, the impact of multiple cultures and trends and the collision of money worship, universal values, Buddhist culture, etc., intertwined with the dregs of traditional culture, have a huge impact on young people. For example, lack of faith and moral decline are no longer uncommon; the proportion of psychological problems and mental illnesses increased; and even frequent psychological crisis events like “depression,” “confusion,” and “anxiety” have become the buzzwords in college campuses, so it is urgent to strengthen the psychological construction, ideological guidance, and value shaping for college students [4–7]. Mental health education and ideological and political education are closely related, the former is an important part of the latter, and the effectiveness of the latter cannot be achieved without the promotion of the positive results of the former. Therefore, from the perspective of integration, it is important to deeply understand the rich connotation of the mental health education curriculum of college students' ideology and politics and reform the curriculum design and teaching practice by setting clear integration teaching objectives, following certain implementation principles, reasonably planning teaching contents, choosing appropriate teaching methods, improving assessment methods, giving full play to the role of the main channel of classroom teaching, and realizing the organic role of psychological education and core values leadership. The integration of psychological education and core values is of great practical significance for both internal and external talent cultivation and for comprehensive development of morality and talent. It not only promotes the realization of the “three comprehensive” education requirements, but also accelerates the development of “greater thinking and politics.”

The schematic diagram of psychology and civics teaching in higher education is shown in Figure 1. Theoretically, it solves the contradiction of “two skins” between civic theory and professional education, clarifies the orientation of education in practice, and unifies the direction of socialist talent training. Reflecting the essence of higher education, the 18th National Congress of the Party has made it clear that “establishing morality and educating people” is the fundamental task of education, establishing morality is the prerequisite and requirement of educating people, and educating people is the goal and value of establishing morality [7, 8]. Moral education is the foundation of colleges and universities, and it is the way to inherit the spirit of Chinese nation and to run a good socialist education with Chinese characteristics. Curriculum Civics requires the role of the main channel in the classroom to urge students to make the core socialist values a guideline to lead their external behavior. By establishing a correct outlook on life, worldview, and values, students can realize a higher sense of value effectiveness and eventually become socialist builders and successors with equal emphasis on competence and moral conduct. The implementation of the concept of “three comprehensive education” is the key to building a system of thinking and education. The Ministry of Education has promoted the construction of two batches of pilot units of comprehensive reform, and although there has been great progress, there are still some problems [9]. The phenomenon of emphasizing the teaching of professional knowledge and skills while neglecting the cultivation of personality and the guidance of values in the teaching of different disciplines still cannot be ignored. The introduction of Curriculum Civics has clarified the mission of professional teachers to educate people and the responsibility of leading values in the classroom, prompting teachers of each course to “guard a section of the canal and plant a responsible field,” to do their duty and work together to realize the essence of education, and further highlight the systematic and holistic nature of ideological and political education. Setting clear teaching objectives is the direction of classroom teaching; the course should be able to effectively support the training objectives, in line with the school's positioning, and talent training objectives. The main contributions of this paper are as follows: (1) Firstly, we assume that the objectives of the civics course should be integrated with the original teaching objectives of the course, and the teaching objectives of the chapter should also be reflected specifically, so as to maximize the civics education function of the mental health education course. In this way, the mental health education course can serve to improve the psychological quality of college students to the greatest extent, and help them to form good psychological quality, so as to realize the education concept of “establishing morality and educating people.” (2) In order to effectively identify the state categories of college students' psychology and civics and fully consider the emotional factors between teachers and college students, this paper proposes a psychological civics teaching model based on graph convolutional neural network. This paper uses Bi-GRU to extract text feature vectors and proposes to use graph convolutional neural network (GCN) for text emotion recognition in psychology and civics teacher-student dialogs, fully considering the emotional interactions between the people involved in psychology and civics teacher-student dialogs, combining two kinds of contextual information to obtain better text representations, and finally for text emotion classification. (3) The obtained experimental results prove that, compared with current classification methods, Bi-GRU combined with GCN model has better performance in sentiment classification.

## 2. Related Work

### 2.1. Teaching Psychology and Civics in Higher Education

Only through the mutual integration of knowledge and value can we realize the comprehensive development of individuals and the sustainable progress of society. In education and teaching, we should not only pay attention to the implicit value leadership in knowledge dissemination, but also emphasize the cohesion of knowledge underpinning in value dissemination, which is also the essence of curriculum thinking and government. Some teachers at college students' mental health education come from the counseling team, are easily influenced by the value neutrality of counseling, and are even confused. However, it should be clear that Curriculum Civics is not psychological counseling; “moral education” itself has ideological attributes; adhering to the correct political direction is necessary; cultivating socialist builders and successors with firm ideals and beliefs is the purpose, so the value leadership here is to serve the goal of talent training; there is a difference between right and wrong [10]. In conclusion, the integration of subject knowledge, competence, and correct value leadership is one of the basic principles that needs to be followed in Curriculum Civics.

Combining explicit teaching and implicit transmission in the classroom helps individuals unknowingly gain experience and influence subsequent behavior in contact with the environment. This requires teachers to pay attention to their own speech and behavior and to infect students with their personality and cultivation. Assisting in problem solving and promoting psychological experience combined with the vigor of college students, in addition to a lot of problems, such as academic delays, information selection difficulties, Internet addiction, interpersonal tension, and out-of-control emotions, to help students solve problems are also part of good ideological and political education. Problem solving is the process of solving a problem through various thinking operations caused by a certain situation and according to a certain goal [11]. Experience is a fusion of emotion-centered sensibility and rationality, and strengthening the psychological experience of successful problem solving can effectively raise the level of individual self-esteem. The formation of virtue is the fusion of the subject and object of the individual's external “situation-event” and internal “experience-experience.” Therefore, the combination of helping individuals to solve problems and promoting psychological experiences can not only achieve the unification of perceptual awareness and rational discernment, but also balance the observational and experiential selves and effectively promote the formation of individual virtues [12–14].

Integration is the most significant feature of the curriculum, which refers to the effective integration and logical post-contraction of the curriculum with other disciplines to achieve its political direction, values, and methodological leadership. Therefore, finding the right point of integration is the key to the construction of the content of Curriculum Civics. The generation of psychological problems among college students is since individual worldview and values are not mature and definite enough. Mental health education in colleges and universities should realize the autonomy of students in understanding and value judgment and the development of individual mind and give proper guidance on personality and moral development while keeping some space for students to think and solve problems, so that students can realize their personality and moral refinement in the process of self-examination. The process of self-examination allows students to achieve character and moral refinement. Full media is gradually penetrating our education system; has a certain positive impact on the civic education in colleges and universities, providing a full-media environment for the innovation of modern education technology; and can effectively promote the reform and innovation of teaching strategies, enhance the effectiveness of civic education in colleges and universities, give a positive role to the whole media, break through the limitations of the obsolete education concept, and achieve the ideal effect of education reform [15–18].

Omni-media refers to the role of information dissemination of multimedia such as animation, images, sound, and web pages; with the help of diversified media forms, like TV, radio, audio and video content, magazines, and other communication paths, business integration of multimedia and media forms, and integration of three networks (broadcasting, telecommunication, and Internet) through information network, users receive the integrated information with the help of communication terminals such as TV and computer, breaking through the time and place. Omni-media has the following four characteristics and plays its value with its own characteristics. First, full media achieves maximum information flow integration. The current existence of the Internet has been updated to 5G; in addition, there are a variety of technical support platforms such as WAP, GSM, CDMA, GPRS, and streaming technology and a rich variety of communication tools, in addition to the traditional newspapers and magazines; there are also the network, telecommunications, satellite communications and other carrier tools to achieve the integration of information flow. Second, full media is compatible with traditional media [19–21]. Full media will improve and innovate traditional media, integrate and use diversified forms of media expression, pay attention to the single form of traditional media, and realize the “full” aspect in the “full” media. Third, omni-media focuses on all-round integration; based on traditional media, omni-media realizes the integration with network media, comprehensive interaction, complementarity, mutual dissolution, and full coverage of omni-media in the information age. This mainly involves the media carrier and audience dissemination of the whole media. Fourth, in addition to the “full” characteristic, it also has the “large” characteristic and provides segmentation services for a wide range of audiences. In the media market, with the help of the omni-media platform, rich forms of information are expressed, and information media are screened according to the different needs of the audience, so that information interaction can be achieved. Full media is built based on “cross-media,” and with the use of media streams, more economical information delivery is achieved, with the outstanding advantages of low investment and good results. Establish the thinking of “Internet + psychological education + curriculum thinking,” break the time and space limitations of the classroom, and build a mixed teaching mode online and offline. The use of online multimedia with images, sound effects, and animations can stimulate students' interest in learning and expand the integration path of learning resources; the equality and interactivity of online communication can effectively stimulate the role of educated subjects and provide a new teaching ecology. In addition, the flipped classroom changes the status of teachers and students in teaching activities and improves the enthusiasm and initiative of students' participation.

### 2.2. Exploring Educational Reform Paths

The classroom is designed to enhance the development of independent thinking and creative thinking by increasing the proportion of discussion and practice among students. The value orientation of the curriculum of “seeing things but not people” will aggravate the dichotomy of knowledge transfer and value guidance and deviate from the fundamental task of “cultivating people” [22]. It is crucial to choose appropriate classroom teaching methods based on the psychological rules of students, the realities of classroom teaching, and the achievement of course objectives. To increase the proportion of student discussion and practice, to enhance the development of independent thinking and creative thinking, and to appropriately reduce the proportion of traditional lectures are an important part of the curriculum reform. Schools that are in a position to do so can conduct small classes where students hold group discussions and become course participants along with the instructor, which can greatly stimulate students' interest in learning. Throughout the process, students are guided to comprehend, practice, and internalize socialist core values at all times through online submission of ideas, classroom group discussions, off-class practical assignments, social research, and other activities, so that individual understanding and practice are mutually evidenced and promoted to achieve unity and recognition of the 3 aspects of socialist core values: rationality, emotion, and behavior. The dual interactive learning path of online knowledge transfer, psychological test, knowledge quiz, group discussion, teacher feedback and expansion, offline case and video sharing, practical activities, teacher and student sharing, value leadership is realized. In addition, the recent emergence of virtual reality technology has enabled the completion of operations that were not possible in teaching in the past. The use of virtual technology can be explored in future course construction, for example, a chapter on emotion management can have different simulation scenarios for students to choose from, that is, public speaking, group discussions, and interviews, to promote the practice of managing students' anxiety in special situations, so that theory and practice can be seamlessly integrated in a relatively short period of time to enhance the effectiveness of the course. This requires teachers to set up new educational thinking, to enrich and update the teaching content as necessary, to introduce content that is in line with the spirit of the times and has a cutting-edge atmosphere, so that students can fully understand and master the essence of the subject. In the process of education and teaching, we can delete the old and outdated contents from the textbooks and introduce the contents that are in line with the spirit of the times and the cutting-edge contents, and we should evaluate the textbooks together with students. At the same time, it is necessary to teach students multiple types and aspects of knowledge in order to facilitate the cultivation of innovative talents. In the process of teaching, teachers need to conduct in-depth research on different versions and different content systems and also need to fully understand the frontier topics of subject development, which should be compared, optimized, analyzed, and organized to reflect the development trend. In terms of teaching content, it is necessary to achieve vigorous reform, innovative teaching content, and dynamic integration with the development of the discipline. Teachers need to teach students not only theoretical and fundamental knowledge, but also to reveal the laws of the discipline, to integrate the theoretical system of the discipline with the social reality, and to keep pace with the development of the times. At present, a big part of the problem is not only the outdated content, but also the repetition and fragmentation of course content, and there is a divergence between knowledge generation processes and knowledge research methods. Teachers need to introduce students to the appropriate background knowledge and always provide the necessary penetration of the scientific method and scientific thinking based on subject knowledge [23]. In addition, it is necessary to ensure that education and teaching are close to real life and reflect the latest achievements of current scientific and technological development. In the process of teaching content innovation and reform, the relevant staff is required to start from the following aspects: First, the staff needs to fully grasp the combination point between major disciplines and also needs to achieve mutual integration, crossover, and communication between disciplines, to achieve the necessary penetration between disciplines, to guarantee students' complete mastery of knowledg. Second, necessary measures need to be taken to enhance students' independent thinking ability and also to further enhance their learning ability. Third, students' scientific thinking should be cultivated. Education is not only about teaching students to apply knowledge, but also about making students investigate knowledge, making them understand the process of knowledge formation, and cultivating their creative spirit and innovative consciousness. In addition, in the process of teaching exercises, teachers are required to dig deeper into the scientific methods embedded in them and to train students in the necessary thinking methods. The whole teaching process needs to penetrate and integrate innovative ideas, pay attention to the cultivation of students' innovative consciousness, guide students to make the necessary discoveries for classroom problems, let students learn to think independently about the problems, and also let students master professional knowledge and then contact scientific research experiments. The key is to cultivate students' innovative thinking, humanistic quality, and practical hands-on ability and guide students to achieve all-round development. In addition, teachers are required to create appropriate teaching situations, cultivate students' innovative spirit, carry out inquiry-based teaching, organize and purposeful teaching activities, guide students to think deeply, cultivate students' interest in innovation, stimulate students' passion for independent inquiry and independent learning, and make students more active and positive in the process of knowledge construction. At the same time, teachers should pass on to students the spirit of rigor and good governance, which is of great value and significance to the cultivation of students. Against the background of innovative talent cultivation, the reform of university education should change the teaching concept, reform the teaching content, and enrich the teaching mode, so that the students' innovative thinking ability and innovative consciousness can be improved. In addition, always adhere to the concept of tolerance, equality, and democracy; encourage students to actively participate in teaching discussions and teaching research; allow students to be different, make mistakes, and say wrong things; and fully respect and understand students. The key is to guide students, not just to instill knowledge into them or adopt a fill-in-the-bag teaching style that is not qualitatively effective and does not improve students' creative thinking and innovative abilities.

## 3. Methods

### 3.1. Model Architecture

The main results of the model are as follows: Bi-GRU is used to extract the sequential contextual features of the psychological and civics teacher-student communication texts; then, a directed graph is constructed with the psychological and civics teacher-student dialog utterances in sequence, and GCN extracts the speaker-level contextual encoding features by aggregating the information of local neighbor nodes; finally, the two different feature vectors are combined for sentiment classification [24–26]. The key to modeling inter-speaker dependencies is the speaker information, which enables the model to understand how speakers affect the emotional states of other speakers. In addition, speaker's own or self-dependence helps to understand the emotional inertia of individual speakers, due to which speakers resist the influence of external factors on their own emotions. Moreover, the relative position of the target discourse and the contextual discourse determines how previously spoken words influence future discourse. The framework of the sentiment recognition method for psychological and Catholic teacher-student dialogs in this paper is broadly divided into 3 parts, as shown in Figure 2, which are a sequence context encoder, whose role is to extract sequence contextual information from the text of dialogs; a speaker-level context encoder, which is used to extract speaker-related contextual features from the dialogs; and a sentiment classifier, which is used to extract speaker-related contextual features from the dialogs by combining the two contextual feature representations and using a similarity-based attention mechanism to obtain the final utterance feature representation, which is input to the fully connected layer for sentiment classification.

### 3.2. Sequential Context Encoder

Suppose we construct a dialog between teachers and students of psychological and ideological teaching, and count the number of people involved in the dialog as *X*, denoted as *e*_1_, *e*_2_,…, *e*_*X*_, and these *X* people say a total of *Y* statements in the dialog, denoted as *u*_1_, *u*_2_,…, *u*_*Y*_. *u*_*t*_ ∈ *R*_*Y*_^*D*^ is the initial feature vector representation, *u*_*t*_ corresponding to the speaker is *es*, and *s* is a mapping between the discourse and its corresponding speaker index. The goal of text sentiment analysis of psychological and ideological teacher-student dialogs is to predict the psychological and ideological teaching status category corresponding to each discourse in the dialogs. In this paper, we use Bi-GRU to extract the textual information features of psychological and civics teacher-student dialogs to obtain the sequential contextual representations of the dialog sentences, and the process is shown in the following equation:

(1) $$\begin{array}{c} \overset{⟶}{g_{t}}=\overset{⟶}{\text{GRU}}\left(\overset{⟶}{g_{t-1}},u_{t}\right),\\ \overset{\leftarrow }{g_{t}}=\overset{⟶}{\text{GRU}}\left(\overset{⟶}{g_{t+1}},u_{t}\right),\\ g_{t}=\left[\overset{⟶}{g_{t}},\overset{\leftarrow }{g_{t}}\right],\;t=1,2,\ldots ,Y\text{,} \end{array}$$

where *u*_*t*_ is the initial context-independent discourse representation; *g*_*t*_ are the outputs of positive GRU and negative GRU, respectively; and *g*_*t*_ is the discourse representation containing the sequence context information. Two unidirectional and opposite directional GRUs form the Bi-GRU network model, and the outputs are jointly determined by the states of the two different GRUs. The specific structure of Bi-GRU is shown in Figure 3.

### 3.3. Speaker-Level Context Encoder

In order to effectively obtain the speaker-level contextual information in the dialog sequences of psychology and civics teachers and students, this paper constructs a directed graph to portray the emotional interactions between psychology and civics teachers and students and uses a spatial domain-based graph convolutional neural network model to obtain a textual representation containing speaker-level contextual information, and the specific structure of the speaker-level context encoder is shown in Figure 4.

A directed graph *G* = {*V, E, R,W*} is constructed to represent the dialog between teachers and students in psychology and civics teaching, where *V* denotes the set of nodes; *E* denotes the set of edges; each discourse is represented as a node *V*_*t*_ ∈ *V*, *t* = 1,2,…, *YV*_*t*_ ∈ *V*, *t* = 1,2,…, *Y*; the initialized feature vector representation is noted as *g*; the edges in node *v* and node *v* are denoted as *r*_*ts*_ ∈ *E*; *r* ∈ *R* denotes the edge relationship type; and the relationship type of the edge depends on two aspects of speaker category and discourse temporal order, i.e., the speaker *es* corresponding to *v* and the sequence of node utterances *v*. Suppose a dialog between teachers and students of psychology and civics teaching contains only two speakers *e*_*1*_ and *e*_*2*_ and a total of five utterances; then, the entire psychology and civics teacher-student dialog constitutes a directed graph as shown in Figure 4. The edge weights *w*_*ts*_ are set using the attention model based on text similarity; i.e., for each node, the weights of the input edges all add up to 1. Considering the m sentences before and the n sentences after each node statement, the weights of the edges between nodes v are specifically calculated in the following equation:

(2) $$\begin{array}{c} w_{ts}=\text{softmax}\left(g_{t}^{T}W\left[g_{t-m},\ldots ,g_{t+n}\right]\right),s=t-m,\ldots ,t+n. \end{array}$$

In the equation, the softmax function ensures that the sum of the total weights of the input edges in node *v* is 1. The graph convolutional neural network model (GCN) uses a two-step graph convolution operation to convert the speaker-independent node by aggregating the local neighbor node feature information of each node feature vector *g*_*t*_ into a new feature vector representation *h*_*t*_ related to speaker information using a two-step graph convolution operation, which is calculated as shown in the following equations. The sum of the total weights of the input edges innode *v* is 1.

(3) $$\begin{array}{c} h_{t}^{\left(1\right)}=\sigma \left(\sum_{r\in R_{s}\in Y_{i}^{\prime }}\frac{w_{ts}}{c_{t,r}}W_{r}^{\left(1\right)}g_{s}+w_{t}W_{0}^{\left(1\right)}g_{t}\right),i=1,2,\ldots ,Y,\\ h_{t}^{\left(2\right)}=\sigma \left(\sum_{s\in Y_{i}^{\prime }}W^{\left(2\right)}h_{s}^{\left(1\right)}+W_{0}^{\left(2\right)}h_{t}^{\left(1\right)}\right),t=1,2,\ldots ,Y. \end{array}$$

### 3.4. Emotion Classifier

The structure of the sentiment classifier is as follows: firstly, the feature vector *g*_*t*_ containing the sequence contextual information and the feature vector *h*_*t*_ related to the speaker information are connected; then, the new psychological and civics teacher-student dialog text feature representation is obtained by the similarity-based attention mechanism; and finally the sentiment classification of the discourse is performed using the fully connected layer psychological and civics teacher-student to get the text corresponding to the psychological and civics teaching state category labels. The connected text vector representations are converted into the final psychological and civics teacher-student dialog text feature representations *h*_*t*_ using a similarity-based attention mechanism.

(4) $$\begin{array}{c} h_{t}=\left[g_{t},h_{t}^{\left(2\right)}\right],\\ \beta_{t}=\text{softmax}\left(h_{t}^{T}W_{\beta }\left[h_{1},\ldots ,h_{Y}\right]\right),\\ {\tilde{h}}_{t}=\beta_{t}{\left[h_{1},\ldots ,h_{Y}\right]}^{T}. \end{array}$$

Finally, the new utterance feature representation *h*_*t*_ is input to the fully connected layer, and the softmax layer performs multi-categorization of the sentiment of text utterances to obtain the maximum probability sentiment label *x*_*t*_.

(5) $$\begin{array}{c} l_{t}=\text{ReLU}\left(W_{1}{\tilde{h}}_{t}+b_{l}\right),\\ X_{t}=\text{softmax}\left(Wl_{t}+b\right),\\ x_{t}=\underset{m}{\text{argmax}}\left(X_{t}\left[m\right]\right). \end{array}$$

## 4. Experiments and Results

### 4.1. Experiment Setup

The specific configuration is shown in Table 1. The experimental dataset selected for this paper's experiments is a crawl through a large number of learning websites of psychology and civics teacher-student dialog. The original data contains about 11318 psychology and civics teacher-student dialogs. The selected part of the corpus was translated into Chinese and used for Chinese psychology and civics teacher-student dialog sentiment analysis research. The excerpted Chinese corpus contains about 600 dialogs between teachers and students in psychology and thinking and political science teaching, with an average of 10 rounds, about 6000 sentences, and 7 categories of psychology and thinking and political science teaching states, namely, neutrality, anger, disgust, fear, happiness, sadness, and surprise. The corpus selected in this paper mainly consists of multiple rounds of psychological and civic studies teacher-student dialogs between two people in daily chat scenes, which involve many relatively rich life topics and extremely rich emotional information, being suitable for psychological and civic studies. The text data are classified, and the corresponding psychological and civics teaching status category labels are obtained. The model hyperparameters are set as shown in Table 2.

In text data preprocessing, in general, symbols do not have great significance to the algorithm. In order to reduce noise interference, we first use regular expressions to filter out useless punctuation marks in the text; then use the stuttering word separation library in *Python* to sub-phrase the text in the experimental dataset; and finally, based on the pretrained word vectors, use the Doc2vec tool to vectorize the text and obtain the text utterance. The obtained input sentence vectors will be used for model training in this paper. The training process loss convergence curve and performance improvement are shown in Figures 5 and 6.

### 4.2. Experimental Results

In order to better carry out the algorithm experiments, the length of the input samples is analyzed in this paper. Suppose the maximum value of the sample length of the selected data set is maxL; then, when the sample length is less than maxL, the sample needs to be filled with zero vector operation to make the sample length reach the maximum value, and when the sample length is greater than maxL, the excess part of the sample needs to be discarded and the overlength sample truncated. The selection of the maximum value of the sample length maxL is related to the good or bad experimental results. When maxL is set larger, the sample data zero vector is overfilled, while when maxL is set smaller, the sample data discard too much information; therefore, setting the maxL size may have some influence on the model performance. In this paper, by setting different maxL, we observe and compare the effect caused by the size of maxL on the model performance, the variation of F1 value with sample length is shown in Figure 7, and the differences of experimental results are shown in Table 3.

Observing Figure 7 and Table 3, we can find that when maxL is set less than 100, the F1 value is relatively low, which is due to too much information discarded from the sample data; when maxL is taken as 100, the F1 value reaches the highest point of 79.54%; when maxL is greater than 100, the F1 value is reduced and the model performance decreases; and the F1 value achieves the lowest value when maxL is 175, which is only 63.66%, because when maxL is set too large, the sample data are filled with too many zero vectors, causing interference with the data features.

In constructing the directed graph of contextual statements, there is a constructed edge relationship between the statement node and several statement nodes before and after it. The experiments in this paper show that the size of F1 value varies with the size of the context window on the dataset as shown in Figure 8; the model performance is poor when the window setting is less than 2; and when the window setting value is larger than 2, the performance rises steadily. For the sake of the number of rounds of dialogue between teachers and students in psychology and Civics teaching in the experiment, this paper sets the window size to 5, and the experimental setting window size of 5 is sufficient in this paper.

In this paper, Bi-GRU + GCN is compared and analyzed with CNN, BiLSTM, Bi-GRU, and other models, and the experimental results of sentiment analysis on Chinese corpus are shown in Figures 9 and 10.

Observing the experimental results of each model, we can see that on the dataset, the F1 value is increased by 15.69% compared with the BiLSTM model and 14.87% compared with the Bi-GRU model. Compared with CNN and BiLSTM models, the hybrid model of Bi-GRU combined with GCN has significantly improved the accuracy of text emotion recognition in dialogs between teachers and students in psychology and civics teaching, and the F1 value is as high as 70.61%, so the overall classification performance is better.

## 5. Conclusion

The addition of artificial intelligence provides a powerful boost to the content dissemination and scene application of civics and political science teaching, which makes civics and political science teaching develop in a more accurate direction in many aspects such as portrait, supply, leadership, and evaluation, directly driving the revolutionary changes in the internal elements and external forms of civics and political science teaching and providing powerful kinetic energy for the governance of major real-life problems in ideological and political education. Therefore, the teaching of civics and political science class should embrace new technologies such as artificial intelligence with open arms. At the same time, we also need to maintain sober awareness; even with the infinite empowerment of technology and powerful help, the ideological attributes of the civics class cannot change; its political guidance and ideological leadership of the basic functions must not be weakened by technology; the logical starting point for the use of technology is the human scale; the purpose is to stimulate the teaching of civics class itself to educate people; technology always has to serve the content, to be adapted to the content. The present is better. In this paper, we fully consider the emotional interaction between speakers, use graph convolutional neural network (GCN) to extract text features related to speakers, then use Bi-GRU model to extract text sequence features to connect the two in order to improve the contextual understanding in the emotional analysis of dialog utterances between teachers and students of psychology and civics teaching, and effectively identify the psychology and civics teaching states in the dialog texts of teachers and students of psychology and civics teaching categories. The experimental results prove the effectiveness of the model, which shows good classification effect in the sentiment analysis of psychological and civics teacher-student dialogs compared with other methods. In this paper, the graph convolutional neural network is used for text sentiment classification of psychological teacher-student dialogs, so only the textual information in the experimental dataset is focused on, and the multimodal sentiment recognition needs to be further studied. The accuracy in sentiment recognition was significantly improved, the F1 value was as high as 70.61%, and the overall classification performance was better. In the future, we plan to use convolutional neural networks for state recognition and reform analysis of psychological and civic teaching.

## Figures and Tables

**Figure 1:** Schematic diagram of psychological and political teaching in colleges and universities.

**Figure 2:** Model structure.

**Figure 3:** Bi-GRU structure.

**Figure 4:** Graph convolution structure.

**Figure 5:** Training process loss convergence curve.

**Figure 6:** Training process performance improvement diagram.

**Figure 7:** Effect of maxL value size on F1 value.

**Figure 8:** Effect of window size on F1.

**Figure 9:** Experimental results on the accuracy of different models.

**Figure 10:** Experimental results of F1 for different models.

**Table 1:** Experimental environment configuration.

Python	3.8
Operating system	Windows 10
CPU	i5 6200U
PyTorch	1.0
Matplotlib	3.4.2
SciPy	1.6.3
Tushare	1.2.62
TA-Lib	0.4.24
yfinance	0.1.59

**Table 2:** Model parameter setting.

Hyperparameter name	Hyperparameter value
Word vector dimension	300
Bi-GRU coding layer dimension	300
Number of Bi-GRU coding layers	1
Number of GCN layers	1
GRU decoding layer dimension	600
Number of GRU decoding layers	1
Batch size	20
Learning rate	0.0008
Optimization algorithm	Adam
Weight decay rate	0.0001

**Table 3:** Effect of sample length on experimental results.

maxL	Accuracy (%)	*F*1 value (%)
50	70.71	70.09
75	79.05	70.45
100	79.54	70.61
125	78.93	70.38
150	79.39	70.54
175	72.41	63.66
200	79.39	70.54

## Data Availability

The datasets used during the current study are available from the corresponding author on reasonable request.
